# Progress of Research on the Application of Triple Antibiotic Paste and Hydrogel Scaffold Materials in Endodontic Revascularization: A Systematic Review

**DOI:** 10.1155/2022/3610461

**Published:** 2022-06-27

**Authors:** Jia Zhao

**Affiliations:** VIP Dental Service, Jinan Stomatological Hospital, Jinan 250001, Shandong, China

## Abstract

**Objective:**

To evaluate the application of hydrogel scaffold materials and triple antibiotic paste in endodontic regeneration through literature review.

**Methods:**

An electronic search of the literature published on PubMed, Wangfang database, and CNKI database using the search terms “endodontic regeneration,” “pulp blood flow reconstruction,” “recanalization,” “triple antibiotic paste,” and “scaffold material” was conducted. The searched literature was used for analysis. *Results and Conclusion.* Hydrogels regulate stem cell fates, modulate growth factor release, and encapsulate antibacterial and anti-inflammatory drugs. The triple antibiotic paste is composed of metronidazole, ciprofloxacin, and minocycline, which exhibits promising antibacterial effects and duration at appropriate concentrations, with low cytotoxicity, and effectively promotes the preservation and regeneration of pulp tissues and the formation of dental hard tissues. However, issues such as tooth discoloration and bacterial drug resistance also exist. The present article reviews the progress of research on the application of hydrogel scaffold materials and triple antibiotic paste in endodontic revascularization.

## 1. Introduction

Pulpal periapical disease is a common disease in dentistry [1]. Endodontic disease is very prevalent in China, with conservative estimates suggesting that more than 80% of the population has varying degrees of endodontic disease, mainly due to the low awareness of oral health among the majority of our population [2]. The pulp is located inside the tooth and is surrounded by highly calcified dentin, in the crown, which is also covered by enamel in the outermost layer, and in the root, which is covered by the bone [3]. Therefore, external stimuli should not generally enter the pulp chamber and cause pulp lesions. Pulpitis is most often caused by infection, which mainly comes from deep caries [4]. Etiologically, pulp disease and periapical disease are broadly similar, for example, severe caries can cause pulpitis, which in turn can cause periapical inflammation [5]. Pathologically, most periapical lesions, especially inflammation, are secondary to endodontic disease, and lesion products and bacteria from the pulp can easily spread to the periapical tissue, which in turn can affect the pulp [6], e.g., acoustic infection from the periodontium can cause lesions in the pulp when the lesions reach the root apex.

Pulpal periapical disease is conventionally treated by apical induction molding followed by filling with nonbiologically active material [7]. However, this approach is unsustainable in preserving the living pulp, resulting in fragile and easily fractured teeth after the loss of sensation such as heat and cold [8, 9], which usually leads to extraction of the affected tooth. Endodontic regeneration is a topical and difficult area of research in recent years, and the American Association of Endodontics defines it as “a biological replacement of damaged tooth tissue, roots, pulp-dentin complex, and other structures to form a functional pulp-like tissue” [9]. Current research has led to two alternative options for achieving pulp regeneration; one is pulp blood flow reconstruction and the other is the regeneration of pulp-dentin complexes using tissue engineering principles. With the development of tissue engineering and materials science, scholars have applied tissue engineering to pulp regeneration studies to obtain long-term tooth retention by inducing differentiation of the pulp-dentin complex through allogeneic/autologous/nested stem cell-scaffold-growth factor complexes [10] to repairing damaged pulp tissue and restoring its physiological function. The control of root canal infection and the choice of the scaffold material are both crucial to the success of this approach [11]. The control of root canal infections is as follows: root canal preparation is mainly done by chemical methods to remove infectious material. Existing studies have concluded that infected root canals are primarily a mixture of aerobic and anaerobic bacteria, for which single antibiotic treatment is of poor efficacy; therefore, triple antibiotic paste, first proposed by Sato et al. in 1996, which contains three antibiotic components (metronidazole, ciprofloxacin, and minocycline), provides excellent antibacterial properties, with less irritation and greater penetration, and has been widely used in endodontic regeneration therapy [12]. Scaffold materials: scaffolds play a bridging role in endodontic regeneration, acting as a delivery system to realize the sustained local release of stem cells and growth factors [13]. In recent years, hydrogels have gained popularity among scaffold materials [14], which have a 95% water content, a three-dimensional structure, some toughness, and rheological properties, and can regulate stem cell fate, modulate growth factor release, and load drugs [15].

This study focuses on the investigation and analysis of hydrogel scaffold materials and triple antibiotic paste in endodontic regeneration. The results are as follows.

## 2. Data Overview and Analysis

### 2.1. Hydrogel Scaffold Materials Commonly Used in Endodontic Regeneration

#### 2.1.1. Natural Hydrogels

Collagen-based hydrogels are one of the earliest and most widely used hydrogel scaffold materials of biological origin [16]. Collagen is the main component of the extracellular matrix and the most abundant protein in mammalian tissues. It can be recognized by cells and degraded by proteases secreted by cells, resulting in good biocompatibility and low immunogenicity. Under certain conditions, collagen molecules can form collagen fibers spontaneously and hydrogels in aqueous solvents. However, prior research found that single-component collagen-based hydrogels exhibit unsatisfactory physical properties, weak mechanical properties, and rapid degradation, and natural collagen is often derived from xenobiotics, which may elicit immune reactions.

Hyaluronic acid-based hydrogels: hyaluronic acid is a proteoglycan that forms the extracellular matrix, and due to its richness in hydrophilic groups, it can be chemically modified and chemically cross-linked to form hydrogel materials under mild conditions with excellent biocompatibility [17]. A caseinized hyaluronic acid-based hydrogel, CorgelTM, was developed in 2009, which undergoes gelation upon addition of a hydrogen peroxide initiator and maintains relative stability with resistance to digestion by hyaluronidase. However, studies have reported that hyaluronic acid often contains impurities and endotoxins that may be pathogenic or cause an immune response, which limits its application. No studies have been reported on its application to regenerate dental pulp in animals in vivo.

Chitosan-based hydrogels are deacetylated products of the natural polysaccharide chitin, a polysaccharide composed of randomly distributed N-acetylglucosamine and glucosamine units, which forms chitosan-based hydrogels by physical association or covalent cross-linking and obtains the desired pore size, degree of cross-linking, and solubility precisely. Studies have shown that chitosan-based hydrogels constitute a dexamethasone release system that can modulate the drug release rate and can also be used as a slow/controlled release carrier for a variety of drugs due to their good biocompatibility, biodegradability, and natural antibacterial effects [18, 19], and have been intensively studied and applied in the biomedical field. However, the application of unmodified chitosan is highly restricted because of its compact crystal structure, which hinders its solubility in neutral solutions and most organic solvents.

### 2.2. Synthetic Hydrogels

Self-assembled peptide hydrogels (SAP): in tissue engineering applications, SAP hydrogels feature good biocompatibility and degradability and can build nanoscale scaffolds and slow-release systems [20], which are novel biomaterials that satisfy a variety of needs in tissue engineering. They usually consist of 15–20 amino acids and have a nanoscale matrix structure similar to an extracellular matrix and good physicochemical properties that allow the hardness and viscosity of the hydrogel to be altered by changing the peptide concentration, thus changing the plasticity of the hydrogel. Self-assembled hydrogels formed based on such a structure can be freely designed and modified to deliver biological functions such as cell adhesion, enzymatic degradation, and proangiogenesis. In recent years SAP has been used in the regeneration of a variety of tissues such as the nerves and the spinal cord, but the complex preparation process, high cost, and limited access have limited the popularization and application of SAP hydrogels.

#### 2.2.1. Multicomponent Hydrogels

Decellularized matrix hydrogels: decellularized matrix hydrogels are scaffold materials that have been well studied in the last decade and are more bionic in composition and structure, offering unparalleled advantages and potential [20]. A decellularized matrix is used to remove immunogenic cellular components by various physicochemical methods to maximize the retention of matrix components. Song et al. isolated a decellularized matrix from the pulp of healthy third molars and used it as scaffold material, which facilitated the proliferation of apical tooth papillae stem cells and the differentiation of adult dentin cells. Nevertheless, the preparation of the scaffold material requires the acquisition of a large amount of autologous tissue, which may cause self-inflicted damage. Thus, the majority of such studies were conducted using a heterogeneous or homogeneous decellularized matrix, which may easily induce immune reactions and present risks of disease carriage and transmission.

### 2.3. Composition and Action Characteristics of Triple Antibiotic Paste

#### 2.3.1. Composition of Triple Antibiotic Paste

The triple antibiotic paste is a paste made of metronidazole, ciprofloxacin, minocycline, and wood slip oil [21].

Metronidazole is a highly effective and less expensive drug of the nitroimidazole class, which is strongly potent against various G+, G-, and anaerobic bacteria and mainly targets anaerobic infections to kill specialized anaerobic bacteria. Metronidazole is selectively toxic to anaerobic microorganisms. Upon entry into the bacteria, the nitro group in the drug molecule is reduced by certain redox proteins to highly reactive nitro radicals, which are capable of disrupting the helix structure of deoxyribonucleic acid (DNA), leading to rapid bacterial death. An analytical study showed that the use of metronidazole as an adjunct to nonsurgical treatment of aggressive periodontitis resulted in better clinical outcomes.

Ciprofloxacin is a broad-spectrum antibacterial drug that belongs to the 3rd generation of quinolone drugs, with strong antibacterial activity, is less liable to produce resistance, and can be used in combination with metronidazole and other drugs for root canal disinfection. Ciprofloxacin inhibits DNA-associated substances such as DNA procyclase in the nucleus of bacteria, causing degradation of DNA and thus producing a bactericidal effect. Ciprofloxacin has very strong antibacterial activity against Gram-negative bacteria, but Gram-positive bacteria and most anaerobic bacteria are resistant to ciprofloxacin. Therefore, ciprofloxacin is often used in combination with metronidazole to treat mixed infections to compensate for the limited antibacterial spectrum. In addition, although ciprofloxacin can cause side effects, the drug can be used safely in clinics at low dose effects.

Minocycline, also known as semisynthetic tetracycline and dimethylaminotetracycline, is a broad-spectrum antimicrobial drug, with fewer resistant bacteria, and only a small amount of use can produce a high local drug concentration, with high efficiency and long-lasting effect. Minocycline accompanies the passive diffusion of cell membranes across the outer membrane of bacteria and invades the inner membrane through active transport to reach the surface of ribosomes within the bacterium and inhibit protein synthesis, ultimately leading to bacterial death. Because minocycline tends to cause discolouration of the tooth structure, it has also been studied as a replacement for other antibiotics to form modified TAP.

#### 2.3.2. Characteristics of the Action of Triple Antibiotic Paste

Triple antibiotic paste possesses strong antimicrobial activity, high penetration, low irritation, less cytotoxicity while exerting antimicrobial disinfection, and good biocompatibility to promote pulp regeneration [22]. Currently, the triple antibiotic paste is widely used as an effective root canal disinfection drug in basic and clinical studies of pulp regeneration.

## 3. Application of Hydrogel Scaffold Materials in Endodontic Regeneration

### 3.1. Advantages of Hydrogels

In tissue engineering, how to achieve a uniform distribution of cells in the scaffold after implantation into the scaffold and how to place the scaffold into the site of action are the key issues that remain to be addressed [23], which are particularly important in endodontic regeneration. In recent years, the extensive use of hydrogels in tissue engineering scaffold materials is attributable to the ability of hydrogels to swell sufficiently in water without dissolving. It is formed by the cross-linking reaction of monomers, and the polymer network formed by the hydrogel can bind water, allowing for good biocompatibility and minimizing the risks of inflammatory reactions in tissues. It is structurally similar to the body tissues and the extracellular matrix, and the soft and moist surface will reduce to a great extent the irritation of the material to the surrounding tissues, and has good permeability where water and its water-soluble small molecules can diffuse freely within the hydrogel [16]. As a result, hydrogel materials present an unparalleled advantage over other materials in endodontic tissue engineering.

### 3.2. Hydrogel Scaffold Materials in Endodontic Regeneration

Regulation of stem cell fate: biomaterials in direct contact with stem cells largely influence the behaviour and differentiation fate of stem cells, including the physical and chemical properties of the material. During endodontic regeneration, hydrogel scaffold materials are modified to promote cell adhesion and migration, increase the rate of material degradation, and maximize the induction of stem cell differentiation for endodontic regeneration. Modulation of growth factor release: it has been reported that inadequate blood supply constitutes one of the challenges for pulp regeneration, and that in spite of sufficient dentin-derived growth factors to promote dentinogenic differentiation of stem cells, insufficiency exists to provide vasculogenic differentiation of stem cells. The direct use of growth factors that promote angiogenesis is associated with failure to maintain long-lasting effects due to their short half-life and rapid metabolism in vivo. In a study using a hydrogel scaffold with cell adhesion and matrix degradation, adding a series of growth factors to the hydrogel via heparin binding and encapsulating pulp stem cells in the scaffold material showed better pulp stem cell proliferation and spreading, superior intercellular cluster formation, and collagen secretion.

Loading of anti-inflammatory drugs: hydrogels can absorb large amounts of water to encapsulate therapeutic drugs to prevent their rapid degradation and control the release rate of encapsulated drugs. Numerous studies have reported that self-assembled peptides can mimic the extracellular matrix structure, promote the growth and differentiation of pulp stem cells, and serve as a satisfactory vehicle for the attachment of growth factors. Colombo et al. predicted that self-assembled peptide hydrogels could be a reliable vehicle for the attachment of abscisins, and by adding bioactive scaffold materials, they could achieve the slow release of abscisins, modulate the inflammatory state of the pulp cavity, and regenerate the pulp-dentin complex.

Loading of antimicrobial drugs: after total pulp necrosis, the bacterial biofilm colonizing the root canal wall is difficult to be completely removed due to the complexity of the root canal system. A foreign study reported for the first time that injectable nanofiber hydrogel slow-release antimicrobial drugs (triple antibiotic paste) are available to avoid direct contact of high local concentrations of drugs with stem cells around the apical foramen, and its sustained release can provide a relatively sterile microenvironment in the root canal, resulting in more stable pulp regeneration.

## 4. The Efficacy and Deficiencies of Triple Antibiotic Paste

### 4.1. Efficacy

The advantages of the triple antibiotic paste are high antibacterial activity, high penetration, long duration of action, and low cytotoxicity, which facilitate the formation of hard tooth tissues and the continued development of the root. Most of the bacteria in the dentin tubules are anaerobic and are the target bacteria for root canal disinfection. The metronidazole in the triple antibiotic paste kills specialized anaerobic bacteria, and is unassociated with dysbiosis and drug-resistant strains, with no contraindications to the combined application of other antibiotics. Its ineffectiveness against parthenogenic anaerobic bacteria can be compensated by minocycline. Minocycline is effective against both parthenogenic anaerobic bacteria and anaerobic bacteria, with stable efficacy and little damage to adjacent tissues, and promotes regeneration of adjacent tissues. Ciprofloxacin is available in combination with metronidazole and other drugs thanks to its broad-spectrum antimicrobial properties and a good bactericidal effect. Based on the pharmacological properties of the three antibiotics, the combination of the three drugs achieved a good root canal disinfection effect [24].

### 4.2. Deficiencies and Countermeasures

Tooth discoloration: during pulpal vascular regeneration treatment, minocycline chelates with Ca2+ in dentin to form insoluble complexes are deposited in the hard tissues of the teeth resulting in tooth discoloration. Porter et al. found that triple antibiotic paste containing doxycycline resulted in lighter dentin staining than triple antibiotic paste containing minocycline, which can be prevented by presealing the dentin tubules through acid etching bonding to inhibit chelation and avoid tooth staining. Alternatively, the use of an injectable nanofiber hydrogel slow-release triple antibiotic paste to avoid direct contact between the high local concentrations of the drug and the stem cells around the apical foramen is also available for the prevention of tooth discoloration. Moreover, Porter et al. also proposed the replacement of minocycline with double antibiotic paste or with other generic antibiotics such as amoxicillin and cefaclor to reduce dentin staining. Results of previous studies have confirmed that the substitution of minocycline with cefaclor and its application in the teeth of animals obviated tooth discoloration.

Destruction of the dentin surface: the results of several studies have shown that triple antibiotic pastes can significantly reduce the hardness of the dentin surface and induce demineralisation of the dentin surface. Yasen et al. found that triple antibiotic paste had a significantly stronger effect on the root canal wall roughness than sodium hypochlorite solution and calcium hydroxide. The countermeasure may involve the selection of an appropriate concentration of triple antibiotic paste or the use of a drug-laden scaffold to slow-release drugs to protect the root canal and reduce erosion.

Bacterial resistance and drug allergic reactions: given the complexity of microorganisms in the root canal, prolonged use or high concentrations of the triple antibiotic paste may produce resistant strains and lead to reinfection and treatment failure. Allergic reactions to drugs such as urticaria or pruritus have been reported with metronidazole, oral mucosal oedema with ciprofloxacin, and pneumonia or eosinophilia with minocycline. Therefore, bacterial culture, drug sensitivity test, exploration for appropriate triple antibiotic paste concentration, and application length are essential. Drug allergic reactions are mostly associated with systemic medications and uncommon with topical medications, for which dentists should be vigilant to protect the physical and mental health of patients.

## 5. Summary and Perspectives

Research on hydrogel scaffold materials has focused on inflammation control, promotion of blood supply, and mimicking the microenvironment of healthy pulp tissues. In recent years, although hydrogel scaffold materials have made milestones in the study of pulp regeneration, the efficient and stable generation of functional pulp-dentin complexes still needs to be explored. The ideal hydrogel scaffold material should have excellent biological properties in endodontic regeneration, mimic ECM, participate in the release of signaling molecules, modulate the behavior of stem cells, and possess excellent physicochemical properties [25]. In terms of composition, collagen, chitosan, and hyaluronic acid are gel components with beneficial biological properties, and peptide hydrogels are currently at the forefront of research. The investigation of endodontic regenerative scaffolds should further screen hydrogels with different components, properties, and functions for scaffold materials with intracanal application characteristics, which can be injected and formed in situ under mild conditions. Triple antibacterial pastes are highly antimicrobial, penetrate well, are ideally antibacterial at the right concentration, and have low cytotoxicity, while effectively promoting the preservation and regeneration of pulp tissue, and the formation of hard tissue in the dentition. Although challenges remain for its application such as tooth discolouration and bacterial resistance, these can be addressed by incorporating hydrogel scaffold materials such as injectable nanofiber hydrogel slow-release triple antibiotic paste to avoid direct contact between high local concentrations of drug and drug stem cells around the apical foramen, and by providing a relatively sterile microenvironment in the root canal and sustained drug release. Currently, a large amount of clinical data and cases are needed for validation.

## 6. Conclusion

In summary, it is currently feasible to obtain stable endodontic regeneration by using injectable nanofiber hydrogel slow-release triple antibiotic paste. A multidisciplinary combination of biomaterials, biomedicine, and tissue engineering is necessary to achieve functional endodontic regeneration in the future to realize the shift from laboratory to clinical practice.

## Data Availability

The datasets used during the present study are available from the corresponding author upon reasonable request.
